# Platelet-Rich Plasma-Derived Exosomal USP15 Promotes Cutaneous Wound Healing via Deubiquitinating EIF4A1

This article has been retracted.

**DOI:** 10.1155/2021/9674809

**Published:** 2021-08-09

**Authors:** Yan Xu, Ze Lin, Lei He, Yanzhen Qu, Liu Ouyang, Yu Han, Chao Xu, Deyu Duan

**Affiliations:** ^1^Department of Orthopaedics, Union Hospital, Tongji Medical College, Huazhong University of Science and Technology, Wuhan 430022, China; ^2^Department of Orthopaedic Surgery, Shanghai Key Laboratory of Orthopaedic Implants, Shanghai Ninth People's Hospital, Shanghai Jiaotong University School of Medicine, Shanghai 200011, China; ^3^College of Life Science and Technology, Huazhong University of Science and Technology, China

## Abstract

Epithelial regeneration is an essential wound healing process, and recent work suggests that different types of exosomes (Exos) can improve wound repair outcomes by promoting such epithelial regeneration. Platelet-rich plasma (PRP) is known to facilitate enhanced wound healing, yet the mechanisms underlying its activity are poorly understood. To explore these mechanisms, we first isolated PRP-derived Exos (PRP-Exos). Using immortalized keratinocytes (HaCaT cells) treated with PBS, PRP, or PRP-Exos, we conducted a series of *in vitro* Cell Counting Kit-8 (CCK-8), EdU, scratch wound, and transwell assays. We then established a wound defect model *in vivo* in mice and assessed differences in the mRNA expression within these wounds to better understand the basis for PRP-mediated wound healing. The functions of PRP-Exos and USP15 in the context of wound healing were then confirmed through additional *in vitro* and *in vivo* experiments. We found that PRP-Exos effectively promoted the *in vitro* proliferation, migration, and wound healing activity of HaCaT cells. USP15 was further identified as a key mediator through which these PRP-Exos were able to promote tissue repair both *in vitro* and *in vivo*. At a mechanistic level, USP15 enhanced the functional properties of HaCaT cells by promoting EIF4A1 deubiquitination. Thus, PRP-Exos and USP15 represent promising tools that can promote wound healing via enhancing epithelial regeneration.

## 1. Introduction

Chronic wounds are defined as wounds that do not heal appropriately and that persist for three months or longer [1, 2]. Such wounds most commonly arise in the context of diabetes, arterial ischemia, poor venous return, infections, pressure ulcers, or malignant tumors, resulting in pain for the affected patient while also compromising the integrity of barriers that are essential for the prevention of bacterial entry into the human body [3]. As such, chronic wounds can reduce patient quality of life while also imposing a significant economic burden on their families and on society as a whole [4]. There is still a lack of any standard treatments for chronic wounds, although keratinocytes are known to be essential mediators of normal wound healing processes [5, 6]. Targeted efforts to accelerate reepithelialization in the context of wound repair thus represent a key area of ongoing scholarly research.

Platelet-rich plasma (PRP) contains a diverse array of physiologically important growth factors at high concentrations, including transforming growth factor-*β* (TGF-*β*), epidermal growth factor (EGF), platelet-derived growth factor (PDGF), and vascular endothelial growth factor (VEGF) [7, 8]. Some of these growth factors are closely related to the formation of blood vessels, which is an integral process in the context of tissue regeneration. Indeed, VEGF-producing Schwann cells have been reported to accelerate peripheral nerve repair [9]. As such, PRP has shown great promise as an applied treatment capable of mediating various forms of tissue regeneration. The therapeutic application of PRP has been linked to accelerated angiogenesis and reepithelialization, thereby promoting expedited wound healing [10]. The mechanisms whereby PRP can promote such regeneration, however, are unclear. In addition to the abovementioned growth factors, platelets can produce a variety of different extracellular vesicles, including exosomes [11], which are small vesicles that are approximately 100 nm in diameter (range: 40–160 nm). These vesicles have been a focus of intensive research interest in recent years owing to their essential role as mediators of cell-cell communication, shuttling nucleic acids, proteins, metabolites, and other macromolecules between cells such that they hold promise as tools for treating a range of diseases [12–15]. Owing to the unique biological properties of PRP and of exosomes, further research is warranted to establish the ability of PRP-derived exosomes (PRP-Exos) to shape wound healing processes *in vitro* and *in vivo*.

The present study was therefore designed to evaluate the impact of PRP-Exos on epithelial cell function to explore the mechanistic basis for such activity *in vitro* and *in vivo* in the context of wound healing.

## 2. Materials and Methods

### 2.1. Cell Culture

HaCaT cells were purchased from the China Center for Type Culture Collection, Wuhan, China, and were cultured in DMEM containing 10%FBS in a 5% CO_2_ incubator at 37°C. Lipofectamine was used to transfect cells with siRNA constructs (50 *μ*mol/L; GenePharma, Shanghai, China).

### 2.2. PRP Preparation

Mice (*n* = 12) were anesthetized via intraperitoneal injection with 1% sodium pentobarbital, after which blood was collected from the abdominal vena cava into a 1 mL syringe containing 0.1 mL of anticoagulant. The collected blood was transferred into a fresh 1.5 mL tube and stored at 4°C until the collection was completed, at which time samples were spun for 10 min at 100 ×*g* at 4°C. The supernatant and the layer containing the white blood cells were then collected from each tube and transferred to a new tube, leaving the red blood cell pellet undisturbed. In this case, normal plasma is obtained. These samples were then spun again for 10 min at 600 ×*g* at 4°C, after which 3/4 of the supernatant was discarded with the remaining sample being gently mixed to yield PRP.

### 2.3. PRP-Exo Isolation and Characterization

Samples of PRP (1.5 mL) were centrifuged for 30 min at 2,000 ×*g*, after which supernatants were collected and centrifuged for 45 min at 12,000 ×*g* at 4°C, and supernatants were then passed through a 0.45 *μ*m filter membrane, after which they were centrifuged for an additional 80 min at 13,000 ×*g*. Supernatants were then discarded, while pellets were resuspended in PBS and centrifuged for 70 min at 110,000 ×*g*, and the remaining particles were suspended in chilled PBS for subsequent analysis. For transmission electron microscopy analyses, these exosomes were combined for 30 min with osmium tetroxide (4%) at 4°C in a 50 *μ*L volume, after which they were transferred onto a copper grid. Next, 1% phosphotungstic acid was utilized to stain these particles, and a transmission electron microscope (Hitachi, HT-7700) was used for their characterization. A NanoFCM™ instrument (N30E) was used for dynamic light scattering (DLS) analyses. Exosome marker protein expression was assessed via Western blotting. Exosomes collected from each subject (*n* = 12) were examined individually. Exosomes were pooled together for use in subsequent cell and animal experiments.

### 2.4. CCK-8 Assay

HaCaT cells were cultured in 96-well plates (5 × 10^3^) for 24, 48, or 72 h, after which they were treated with the CCK-8 reagent for 2 h (G4103, Servicebio). Absorbance was then measured at 450 nm to assess cell proliferation.

### 2.5. EdU Assay

HaCaT cells were plated in 24-well plates (1 × 10^5^/well) and treated as appropriate for 24 h, after which EdU staining was performed based on provided directions (G1601, Servicebio).

### 2.6. Wound Healing Assay

Following appropriate treatments, HaCaT cell monolayers cultured in 6-well plates were scratched with sterile 10 *μ*L pipette tips to generate linear scratch wounds. Cells were then incubated in the serum-free media for 12 or 24 h, after which they were imaged via inverted microscope.

### 2.7. Transwell Migration Assay

Cells were added to the upper chamber of a Transwell filter with an 8 *μ*m pore size (3 × 10^4^/well) in 200 *μ*L of serum-free media, after which the lower chamber was filled with 600 *μ*L of media containing Exos or other appropriate reagents. Following incubation for 24 h, the number of migratory cells was assessed via light microscopy.

### 2.8. Cell Cycle Analysis

Cell cycle progression was assessed via flow cytometry using a cell cycle and apoptosis analysis kit (G1700; use G1700-50T, Servicebio) based on the provided directions.

### 2.9. Western Blotting

After total protein extraction, 40 *μ*g of protein per sample was separated via 10% SDS-PAGE and transferred to PVDF membranes that were stained overnight at 4°C with primary antibodies, after which they were probed for 1 h with HRP-conjugated secondary antibodies at 37°C. The following antibodies were used: anti-CD9 (1 : 1000, Abcam, ab223052), anti-TSG101 (1 : 1000, Abcam, ab125011), anti-Calnexin (1 : 1000, Abcam, ab22595), anti-USP15 (1 : 500, Abcam, ab71713), and anti-EIF4A1 (1 : 1000, Abcam, ab31217).

### 2.10. Quantitative Real-Time PCR (qPCR)

TRIzol (Invitrogen) was used to isolate total RNA from prepared samples, after which 1 *μ*g of this RNA was used to prepare cDNA. A StepOne™ Real-Time PCR system (Life Technologies, CA, USA) was used to conduct all qPCR reactions, with the 2^−*ΔΔ*Ct^ method being used to assess relative gene expression and GAPDH serving as a normalization control. Primer sequences were as follows: USP15: forward: 5′-AAAACCTCGCTCCGGAAAGG-3′, reverse: 5′-CCACCTTTCGTGCTATTGG-3′; EIF4A1: forward: 5′-TGTCTGCGAGCCAGGATTCCC-3′, reverse: 5′-AGATGCCACGGAGAAGGGACTC-3′.

### 2.11. Murine Cutaneous Wound Model Establishment

Male C57BL/6 male mice (6–8 weeks old) from the Center of Experimental Animals, Tongji Medical College, Huazhong University of Science and Technology, were individually housed in an 18°C facility with a 12 h light/dark cycle. Animals were anesthetized using intraperitoneal pentobarbital sodium with no signs of peritonitis, pain, or discomfort, after which a 10 mm diameter full-thickness excisional skin wound was generated on the dorsum of each animal. Mice were then randomly assigned to five treatment groups that were treated with PBS (100 *μ*L), PRP-Exos (100 *μ*g PRP-Exos in 100 *μ*L PBS), siRNA-NC (in PBS), siRNA-USP15 (in PBS), or siRNA-USP15+PRP-Exos (in PBS). For siRNA-NC and siRNA-USP15 treatments, animals were administered 100 *μ*L of a 20 *μ*mol/L preparation of the corresponding siRNA, while for the siRNA-USP15+PRP-Exos treatment group, mice were administered 100 *μ*L of a 10 *μ*mol/L siRNA preparation and 10 *μ*mol/L of PRP-Exos in PBS. All prepared solutions were injected subcutaneously in appropriate mice at four sites adjacent to the wounded area (25 *μ*L/site). Images of the wounds were captured on days 0, 3, 7, 10, and 14 postwounding. Animals were euthanized on day 14, at which time skin samples were collected for downstream analyses. Wound area was measured with the ImageJ software, and wound healing was calculated as follows: Wound healing = (Wound area on Day *n*/Wound area on Day 0) (Wound area on Day *n*/Wound area on Day 0) × 100.

The Animal Care and Use Committee of the Tongji Medical College, Huazhong University of Science and Technology, approved all animal studies detailed herein.

### 2.12. Hematoxylin and Eosin Staining, Masson's Trichrome Staining, and Immunohistochemical Staining

Paraffin-embedded tissue sections (7 *μ*m thick) were subjected to hematoxylin and eosin (H&E) and Masson's trichrome staining. An immunofluorescent approach was used to detect USP15 in prepared tissue sections. Briefly, prepared sections were blocked for 30 min with 1% BSA, probed overnight with anti-USP15 (1 : 500, Abcam, ab71713), and stained for 1 h with an appropriate secondary antibody, and then, USP15-positive cells area in three random fields of view were analyzed. All stained tissue sections were independently assessed by three observers blinded to experimental treatment protocols.

## 3. Results

### 3.1. PRP-Exo Characterization

Transmission electron microscopy (TEM), dynamic light scattering (DLS), and Western blotting were initially used to characterize isolated PRP-Exo samples. The obtained PRP-Exos ranged from 40 to 100 nm in size (Figures 1(a) and 1(b)), with the majority of these particles exhibiting cup-shaped or spheroid morphological characteristics consistent with those of Exos. Western blotting analyses indicated the presence of the exosomal markers CD9 and TSG101 in these samples (Figure 1(c)), thus confirming the successful enrichment of exosomes from PRP samples.

### 3.2. PRP-Exo Treatment Enhances *In Vitro* Keratinocyte Responses

The impact of PRP-Exo treatment on immortalized human keratinocytes (HaCaT cells) was next assessed. To establish the uptake of these exosomes by HaCaT cells, these particles were initially labeled using the lipophilic PKH26 dye, followed by incubation in cell culture media for 8 h at which time the uptake of these fluorescent particles was clearly evident (Figure 2(a)). HaCaT cells were then treated with PBS, PRP, or PRP-Exos, and their proliferation was assessed through a series of CCK-8 and EdU uptake assays, confirming that PRP-Exo exposure was associated with the enhanced proliferation of these keratinocytes (Figures 2(b) and 2(c)). PRP-Exo treatment was associated with an increase in the frequency of HaCaT cells entering the S stage of the cell cycle (Figure 2(d)). Following PRP-Exo treatment, higher levels of cell cycle-associated proteins were found to be expressed in these cells (Figure 2(e)). In Transwell and wound healing assays, PRP-Exo treatment was also associated with significant improvements in HaCaT cell migration (Figures 2(f)–2(h)). Together, these data thus indicate that PRP-Exo treatment can significantly augment HaCaT cell proliferation and migration.

### 3.3. PRP-Exo Treatment Enhances *In Vivo* Wound Healing in Mice

An *in vivo* cutaneous wound model was next established using C57BL/6 mice, with equal volumes of PBS, PRP, or PRP-Exo preparations being injected around the wound site in each animal to assess the impact of such treatment on wound healing. Relative to control animals, those treated with PRP and PRP-Exos exhibited faster wound repair, with such healing being even more rapid for PRP-Exo-treated mice relative to mice treated with PRP alone (Figures 3(a) and 3(b)). The scars of mice in the PRP-Exo group were smaller than those of mice in any other group (Figure 3(c)), and these mice exhibited the highest levels of collagen formation (Figure 3(d)). Reepithelialization plays an essential role in the wound healing process [16]. Deubiquitinases (DUBs) can alter protein stability by removing a ubiquitin chain from a given protein, thereby stabilizing it [17], thus potentially accelerating the process of reepithelialization in the context of wound healing. The ubiquitin-specific protease (USP) family is the best-studied group of DUB proteins, and USP15 is an important member of this family [18]. As such, we next evaluated the expression of USP15 in keratinocytes in wounded skin tissues, revealing it to be expressed at higher levels in the PRP-Exo treatment group (Figure 3(e)).

### 3.4. USP15 Is Enriched in PRP-Exo Preparations

To explore the functional importance of USP15 as a driver of PRP-Exo-mediated wound healing, we assessed the levels of this protein in PRP and PRP-Exo samples via Western blotting, revealing it to be present at significantly higher levels in PRP-Exos (Figure 4(a)). Subsequent qPCR analyses additionally exhibited increased USP15 expression in PRP-Exos at the mRNA level (Figure 4(b)). Similarly, higher USP15 protein levels were evident in epidermal keratinocytes in the PRP-Exo group *in vivo* (Figures 4(c) and Figure 3(e)), suggesting that USP15 may be linked to the ability of PRP-Exos to promote wound healing.

### 3.5. PRP-Exos Promotes HaCaT Cell Migration and Proliferation in a USP15-Dependent Manner

To understand the functional effects of USP15 on HaCaT cells, they were next treated with PBS, PRP, and PRP-Exos. Western blotting indicated that USP15 levels were highest for HaCaT cells treated with PRP-Exos (Figure 5(a)). As shown in Figure 1, HaCaTs treated with PRP-Exos exhibited significantly augmented cellular proliferation and migration. In contrast, siUSP15 treatment had the opposite effect on HaCaT cell proliferation and migration in these same assay systems (Figures 5(b)–5(e)). As such, decreasing USP15 expression in HaCaT cells can reduce the beneficial impact of PRP-Exo treatment. Together, these findings suggest that USP15 is the primary mediator whereby PRP-Exos promote HaCaT cell migration and proliferation.

### 3.6. USP15 Enhances HaCaT Cell Functionality by Promoting EIF4A1 Deubiquitination

We next explored the mechanisms whereby USP15 promotes HaCaT cell functionality. EIF4A1 is a key eukaryotic initiation factor complex component that has been linked to the proliferation of certain cell lines [19, 20], although it has not been studied in detail in HaCaT cells. As such, we hypothesized that USP15 may be able to promote HaCaT cell proliferation in part via altering the EIF4A1 expression. To examine the effects of USP15 on EIF4A1 stability in HaCaT cells, we conducted Western blotting assays which revealed a significant decrease in both USP15 and EIF4A1 expressions following siRNA-USP15 treatment (Figure 6(a) and 6(b)), whereas qPCR analyses indicated that the EIF4A1 mRNA levels in these cells were unchanged (Figure 6(c)).

We then assessed the functional importance of EIF4A1 in HaCaT cells by knocking down this gene with a specific siRNA construct. Subsequent CCK-8 and EdU assays suggested that EIF4A1 knockdown was sufficient to suppress HaCaT cell proliferation (Figures 6(d) and 6(e)), with Western blotting being used to confirm that EIF4A1 protein levels were reduced following siRNA transfection (Figure 6(f)). In Transwell and wound healing assays, siRNA EIF4A1 treatment significantly reduced the migratory activity of these keratinocytes (Figures 6(g) and 6(h)). Together, these data suggested that USP15 can enhance the migration and proliferation of HaCaT cells by promoting EIF4A1 deubiquitination.

### 3.7. USP15 Promotes Wound Healing *In Vivo*

To examine the impact of USP15 on wound healing processes, equivalent amounts of PBS, siRNA-NC, siRNA-USP15, siRNA-USP15, or PRP-Exos were injected surrounding wound sites in C57/BL6 mice, as above. USP15 knockdown was found to significantly slow the wound healing process in these animals (Figures 7(a) and 7(b)), and H&E staining confirmed that wounds in the siRNA-USP15 group were larger than those in other groups (Figure 7(c)). Masson's trichrome staining also revealed that collagen levels were lowest in the siRNA-USP15 group (Figure 7(d)), and the number of USP15-positive cells in murine wound sites was lower in siRNA-USP15-treated mice relative to other groups (Figures 7(e) and 7(f)). Together, these results thus demonstrated that USP15 knockdown was sufficient to largely ablate the beneficial effects of PRP-Exo treatment in the context of *in vivo* cutaneous wound healing.

## 4. Discussion

A number of clinical strategies have been employed in recent years in an effort to accelerate wound healing [21]. PRP-based therapies have emerged as promising means of promoting wound healing and have been studied in the fields of orthopedics, dermatology, dentistry, and diabetic wound management. However, there have been few studies to date of PRP-Exos. Herein, we determined that PRP-Exo treatment was sufficient to promote wound healing in a manner more efficient than direct PRP treatment. The process of epidermal regeneration is a multistep process that is regulated by a range of cytokine and cell types, ultimately leading to the reconstruction of the damaged skin barrier [22]. Exosomes derived from mesenchymal stem cells have been repeatedly shown to accelerate reepithelialization and to thereby enhance wound healing [23, 24]. Our present results indicated that PRP-Exo treatment similarly promoted enhanced epithelialization, highlighting the promise of these particles for use in the treatment of chronic wounds.

Exosomes are small, lipid bilayer-enclosed extracellular vesicles that are produced by most known cell types and that can transmit macromolecules and other compounds between cells [25]. When taken up by recipient cells, these exosomes can thus alter cellular functionality via the delivery of specific proteins, nucleic acids, and signaling molecules in a manner that makes them ideal for use as drug carriers in a range of disease types [24]. Herein, we found that HaCaT cells were able to efficiently internalize PRP-Exos. It has been reported that a range of new types of hydrogels with specifically tailored biochemical functions can accelerate wound healing, thus exhibiting good prospects for therapeutic application [26, 27]. However, such artificial hydrogels play a less direct role in normal physiological processes, and a combination of exosomes and hydrogels may thus offer greater advantages further expediting the wound healing process.

Protein ubiquitination has been shown to play diverse regulatory roles in the context of wound healing [28, 29]. USP family proteins, including USP15, are key mediators of protein deubiquitination. Others have reported that PRP can promote wound healing by driving accelerated epithelialization [30], and we herein found that PRP-Exo treatment was superior to PRP treatment as a means of enhancing wound healing in a manner associated with increased USP15 protein levels in wound tissues relative to those detected upon PBS or PRP administration. Through a series of *in vitro* and *in vivo* experiments, we further confirmed that USP15 was able to promote wound healing, suggesting that PRP-Exo-derived USP15 is a key mechanism driving this regenerative process. Tao et al. have reported that PRP-Exos can suppress apoptosis in a rat model of femoral head osteonecrosis via the Akt/Bad/Bcl-2 signaling pathway [31], while Iyer et al. revealed the ability of PRP-Exo treatment to promote functional recovery following muscle injury [32]. Owing to their unique properties, exosomes have been shown to be of value for the treatment of many diseases and thus warrant further clinical study.

In prior studies, USP15 was shown to interact with EIF4A1 and to thereby accelerate wound healing [33]. Consistent with such a model, we found that USP15 knockdown was sufficient to reduce EIF4A1 expression, while EIF4A1 knockdown directly impaired HaCaT cell migration and proliferation. Together, these results suggest that the USP15-EIF4A1 axis is a key mediator of the reepithelialization process.

## 5. Conclusion

In conclusion, the results of this study indicate that PRP-Exo-derived USP15 is a key mediator of HaCaT cell survival and migratory activity, with EIF4A1 playing an important role in the process of USP15-induced epithelialization (Figure 8). Together, these findings provide a robust foundation for future studies of the therapeutic potential of PRP-Exo treatment as a means of promoting improved wound healing.

## Figures and Tables

**Figure 1:** PRP-Exo characterization: (a) TEM images of PRP-Exos; (b) PRP-Exo size distributions, as measured via DLS; (c) Western blotting analyses of proteins within PRP-Exos.

**Figure 2:** PRP-Exos enhance HaCaT cell proliferation and migration. (a) HaCaT cells were able to take up PKH26-labelled PRP-Exos. (b, c) CCK-8 and EdU uptake assays were used to assess the impact of PRP-Exo treatment on HaCaT cells. (d) Flow cytometry was used to assess how PRP-Exos affect cell cycle progression. (e) Western blotting was used to assess levels of cell-cycle associated proteins (cyclin D1 and cyclin D3) following PRP-Exo treatment. (f) Wound healing and (g, h) Transwell assays were used to gauge the impact of PRP-Exos on HaCaT cell migration. ^∗^*P* < 0.05, ^∗∗^*P* < 0.01, ^∗∗∗^*P* < 0.001, and ^∗∗∗∗^*P* < 0.0001.

**Figure 3:** PRP-Exos promote wound healing in C57BL/6 mice. (a) Images of wounds in representative mice. (b) Wound healing rates in the control, PRP, and PRP-Exo treatment groups. (c, d) H&E staining and Masson's staining results from the three treatment groups with corresponding quantification results. (e) USP15 immunohistochemistry results for wound sections in the three treatment groups. ^∗^*P* < 0.05, ^∗∗^*P* < 0.01, ^∗∗∗^*P* < 0.001, and ^∗∗∗∗^*P* < 0.0001. *n* = 6.

**Figure 4:** PRP-Exos contain high levels of USP15, which promotes enhanced HaCaT cell functionality. (a) Western blotting was used to assess USP15 levels in PRP and PRP-Exos. (b) USP15 mRNA levels were assessed via qPCR. (c) USP15 levels in murine wound tissues were assessed via Western blotting. Data are from three independent experiments. ^∗^*P* < 0.05, ^∗∗^*P* < 0.01, and ^∗∗∗^*P* < 0.001.

**Figure 5:** USP15 promotes in vitro wound healing. (a) Western blotting data demonstrating USP15 levels in control, PRP, and PRP-Exos groups. (c, e) Wound healing and Transwell assays were used to assess the migratory activity of HaCaT cells. (d) The proliferation of HaCaT cells in the indicated treatment groups was assessed via CCK-8 assay. Data are from three independent experiments. ^∗^*P* < 0.05, ^∗∗^*P* < 0.01, ^∗∗∗^*P* < 0.001.

**Figure 6:** USP15 promotes EIF4A1 deubiquitination to enhance HaCaT cell functionality. (a, b) Western blotting results demonstrating USP15 and EIF4A1 levels in HaCaT cells following siRNA-USP15 treatment. (c) EIF4A1 levels in HaCaT cells following siRNA-USP15 treatment, as assessed via qPCR. (d, e) HaCaT cell proliferation was assessed via CCK-8 and EdU assays following siRNA-EIF4A1 treatment. (f) Western blotting analyses were used to assess EIF4A1 expression HaCaT cells following siRNA-EIF4A1 treatment. (g, h) Wound healing and Transwell assays were used to assess the migratory activity of HaCaT cells following siRNA-EIF4A1 treatment. Data are from three independent experiments. ^∗^*P* < 0.05, ^∗∗^*P* < 0.01, and ^∗∗∗^*P* < 0.001.

**Figure 7:** USP15 promotes in vivo wound healing. (a) Images of mice in the three treatment groups. (b) Wound closure rates for mice in the three treatment groups. (c) H&E staining results from the three treatment groups. (d) Masson's trichrome staining results for wounds in the three treatment groups. (e) USP15 immunohistochemical staining results for the three groups. (f) Quantification results for data in the three treatment groups. ^∗^*P* < 0.05, ^∗∗^*P* < 0.01, ^∗∗∗^*P* < 0.001, and ^∗∗∗∗^*P* < 0.0001. *n* = 6.

**Figure 8:** USP15 is one of the main mRNA in PRP-Exos, which could be taken into HaCaTs, subsequently deubiquitinating EIF4A1, then accelerating reepithelialization and promoting wound healing.

## Data Availability

Data available on request.
